The article "Management of Malpositioned Cervical Interfacet Spacers: An Institutional Case Series" was published in 2021. Journal: Cureus.

# Management of Malpositioned Cervical Interfacet Spacers: An Institutional Case Series

**DOI:** 10.7759/cureus.20450

**Published:** 2021-12-15

**Authors:** Joseph H Garcia, Alexander F Haddad, Arati Patel, Michael M Safaee, Brenton Pennicooke, Praveen V Mummaneni, Aaron J Clark

**Affiliations:** 1 Neurological Surgery, University of California San Francisco, San Francisco, USA

**Keywords:** interfacet spacer, malposition, cervical spondylosis, cervical radiculopathy, cervical myelopathy

## Abstract

Introduction

Posterior cervical foraminotomy and anterior cervical discectomy and fusion (ACDF) are the mainstay treatments for cervical radiculopathy. A recent alternative or adjunct involves the placement of interfacet spacers, which promote indirect decompression by increasing foraminal height. Cervical interfacet spacers have been shown to be safe options for indirect decompression and improve short-term clinical outcomes in patients with cervical spine pathologies. However, no previous data regarding malpositioned spacers and their management have been reported. Given this paucity of data, we aim to present examples of malpositioned interfacet spacers and their management.

Methods

This was a retrospective single-center review.

Results

Twenty-five patients were identified in which interfacet spacers were used at a single level in 19 cases, two levels in five cases, and three levels in one case. The cohort had a mean follow-up of 14.4 months. Among 60 total spacers placed, two required repositioning (3.3%). The first underwent bilateral placement at C4/5 and developed a unilateral deltoid palsy postoperatively. She was taken back to the operating room the same day for implant removal. A second patient underwent removal after a malpositioned implant at C4/5 was identified on an intraoperative CT scan. A third patient had spacers placed at a referring hospital and presented with progressive neck pain and radiculopathy. She underwent successful removal with a resolution of her symptoms.

Conclusions

Interfacet spacers represent a novel technique for the treatment of cervical radiculopathy, however, there are limited data on their utilization. We present the first reports of malpositioned spacers and their management. Patients with small facet joints and lateral masses may be at increased risk for malposition, and intraoperative fluoroscopy may not adequately confirm implant placement. Surgeons should use caution when implementing new technology with a low threshold for intraoperative CT to confirm the appropriate placement of these devices.

## Introduction

Posterior cervical decompression and fusion (PCF) is a mainstay of treatment for cervical spondylotic myelopathy, one of the most common adult spinal disorders in the United States (US) [1-2]. Lateral mass screw fixation and laminectomy are standard techniques for PCF, however, patients with radiculopathy require additional foraminotomies or anterior cervical discectomy and fusion (ACDF) to address nerve root compression.

Cervical interfacet spacers are a recent addition to the surgeon’s armamentarium. These devices are designed to provide indirect decompression of cervical nerve roots by increasing neuroforaminal height (DTRAX® Cervical Cage, Providence Medical Technology; Lafayette, CA, and FacetLift, Medtronic; Minneapolis, MN). They are placed through a traditional posterior approach and carefully inserted into the facet joint after decortication in order to promote fusion [3]. Early clinical results are encouraging, however, additional studies are needed to determine the efficacy and long-term outcomes associated with this technique compared to traditional procedures, including lateral mass screw fixation with foraminotomies or ACDF [3-5].

We present our comprehensive institutional experience with the use of cervical interfacet spacers placed through a traditional open posterior approach. Cases were reviewed to identify postoperative neurologic deficits or symptoms directly attributable to malpositioned cages that subsequently required surgical revision.

## Materials and methods

Patient identification

Adult patients undergoing interfacet spacer placement from 2016-2019 were identified through a retrospective review of surgical records at a single academic medical center. All patients had these devices placed through an open posterior cervical approach as an adjunct to their instrumented fusion. Individual patient consent was not required given the study design - retrospective chart review with no patient contact or use of identifying information. Research activities were performed under the Committee on Human Research (CHR# 19-29440), our Institutional Review Board. Medical records and operative reports were reviewed to identify cases in which interfacet spacers had to be repositioned or cases that resulted in a postoperative neurologic deficit or other complication. All surgeries were performed by fellowship-trained spine surgeons.

## Results

Institutional experience

Twenty-five patients who underwent PCF with the use of interfacet spacers at our institution were identified. The mean age was 60 years with 12 women (48%). Spacers were used at a single level in 19 cases, two levels in five cases, and three levels in one case. In certain cases, spacers were only placed unilaterally. The number of instrumented levels were as follows: 12 C1/2, 1 C2/3, 7 C3/4, 20 C4/5, 13 C5/6, and 7 C6/7, for a total of 60 implants. A graphical representation of instrumented levels is shown in Figure 1. Spacers used at C1/2 were primarily used to promote arthrodesis rather than indirect decompression. Two implants (3.3%) required revisions as described below. These were the only cases associated with a new neurologic deficit or perioperative complication related to interfacet spacer placement. Both cases involved spacers inserted at the C4/5 level and resulted in mild postoperative deltoid palsies. A summary of postoperative neurologic exams by implant level is shown in Table 1. The cohort had a mean follow-up of 14.4 months.

**Figure 1:** Interfacet spacer level distribution A total of 25 patients underwent placement of 60 interfacet spacers as shown above.

**Table 1:** Postoperative neurologic exams by interfacet implant level Exams were defined as either improved/stable or worse compared to preoperative exams.

DTRAX Level	Motor Exam Stable/Improved	Motor Exam Worse
C1-2	12	0
C2-3	1	0
C3-4	7	0
C4-5	18	2
C5-6	13	0
C6-7	7	0

Case 1

A 74-year-old woman presented with neck pain, gait instability, and urinary incontinence. MRI demonstrated severe stenosis from C2-C6 with associated cord signal change and bilateral foraminal stenosis at C4-C5. She was taken for C2-C6 laminectomies and instrumented fusion with left C3/4 and bilateral C4/5 interfacet spacers. Intraoperative motor evoked potentials (MEP) and somatosensory evoked potentials (SEP) were stable throughout the case. Postoperative exam demonstrated mild right deltoid and bicep weakness with a postoperative CT showing neuroforaminal stenosis at C4-5 (Figure 2). An MR neurogram was obtained and demonstrated normal course, caliber, and signal intensity of the brachial plexus. She was taken back to the operating room the same day for removal of the right interfacet implant and foraminotomy. Her hospital course was otherwise uncomplicated, and her deltoid and bicep strength were normal at the 12-month follow-up.

**Figure 2:** Case 1 – Malpositioned C4/5 interfacet implant Immediate postoperative axial CT (A) shows impingement of the right C4/5 neural foramen by a medialized interfacet spacer (arrowhead). Coronal (B) and sagittal (C) CT images confirm impingement of the interfacet spacer on the right C4/5 neural foramen.

Case 2

A 69-year-old woman with a history of T7-T8 instrumented fusion and 12 months of gait instability presented with acute worsening of gait and new urinary incontinence. MRI demonstrated C3-C7 stenosis with underlying cord contusion. She was taken to the operating room for C3-T1 instrumented fusion with C4-C7 laminectomies, foraminotomies, and bilateral C4/5 interfacet spacers. Intraoperative neuromonitoring was notable for a 70% decrease in MEPs of the right deltoid and biceps after placement of the interfacet implants. Intraoperative CT showed that the right implant was impinging on the foramen and was therefore removed (Figure 3). The postoperative exam was notable for mild deltoid palsy that was resolved by a six-week follow-up visit.

**Figure 3:** Case 2 – Malpositioned C4/5 interfacet implant with intraoperative removal The intraoperative CT scan demonstrates a medialized right C4/5 interfacet spacer causing impingement of the neural foramen (A). The malposition was recognized and the interfacet spacer was removed. A second intraoperative CT scan demonstrated resolution of foraminal stenosis at that level (B).

Case 3

 A 57-year-old woman with a remote non-instrumented C5/6 anterior cervical discectomy and fusion presented with progressively worsening neck pain after undergoing placement of bilateral C3/4 and C4/5 facet implants 12 months prior at a referring facility. Imaging demonstrated facet spacers at the C3/4 and C4/5 levels with associated foraminal stenosis at both levels on the left side (Figure 4). Her case was presented at our multi-disciplinary spine conference that included neurologists, neuroradiologists, and neurosurgeons specializing in spine surgery. The consensus was that although the foraminal stenosis was not causing obvious symptoms involving the C4 or C5 nerve roots, her worsening neck pain and severe radiographic stenosis warranted removal of these implants followed by C3-C5 lateral mass screw fixation.

**Figure 4:** Preoperative and postoperative imaging after removal of malpositioned interfacet implant Axial CT at C3/4 (A) and C4/5 (B) demonstrate implant impingement along the left C4/5 foramen. Sagittal CT along the left (C) and right (D) cervical facets demonstrate impingement of the left C3/4 and C4/5 neural foramen. Postoperative anteroposterior (E) and lateral (F) X-rays demonstrate the successful removal of interfacet implants with the placement of lateral mass fixation from C3-C5 bilaterally.

She was taken to the operating room for the aforementioned procedure. Exposure of the C3-C5 lateral masses was achieved through a traditional midline posterior approach. There was bone overlying the C3/4 and C4/5 facets, however, the joints were clearly mobile, consistent with pseudarthrosis. A high-speed burr was used to drill the facets a few millimeters lateral and medial to the implant, as well as a few millimeters above and below. Since the implant included a screw embedded in the lateral mass, a Penfield #4 dissector was used to gently distract open the facet joint while the implant was grasped using a needle-nose Leksell and gently rocked lateral to medial and craniocaudally to facilitate removal (Video 1). Lateral mass screws were placed from C3 to C5 and secured to a rod. The facets and posterolateral spine were packed with bone graft. The patient was discharged home on postoperative day 3 in good condition. At the three-month follow-up, she reported improvement in her neck pain with cervical X-rays demonstrating normal implant alignment.

**Video 1:** Intraoperative removal of interfacet spacer Technique demonstrating removal of a malpositioned cervical interfacet spacer.

## Discussion

Cervical interfacet spacers represent a novel strategy for the treatment of symptomatic cervical radiculopathy. We present our institutional experience with the use of these devices. The rate of malposition was 3.3%, which is similar to or less than revision rates found in single-center ACDF or PCF series with equivalent patient follow-up [6-7]. In all cases, implants were revised without complication. Two patients in our cohort had a worse neurologic motor exam postoperatively. Interestingly, both were deltoid palsies after C4/5 interfacet spacers. This is consistent with the C5 nerve root being the most sensitive to stretch and neuropraxic injury after posterior cervical surgery [8]. Although the precise factors that predispose C5 to postoperative palsies are unclear, prior case series have identified ossification of the posterior longitudinal ligament and decreased foraminal diameter as risk factors for deficits following surgery [9-10]. In any case, these results indicate that additional caution should be taken when placing C4-5 spacers.

By distracting the facet these devices, have the potential to provide indirect decompression of symptomatic levels by increasing neuroforaminal height. Goel and Shah validated facet distraction as a strategy for treating symptomatic cord and nerve root compression in 36 patients. Four subsequent cadaveric studies found that foraminal height and area were significantly increased with spacers [11] and associated with significant reductions in range of motion, however, a careful review of these data suggest that lateral mass screws are associated with a less segmental range of motion compared to interfacet spacers, particularly in flexion-extension [12].

Preliminary results in 60 patients were presented by McCormack et al. in 2013 [5]. At the one-year follow-up, mean Neck Disability Index (NDI), Short Form 12 item (version 2) (SF-12v2), and visual analog score (VAS) scores were significantly improved. Segmental lordosis at treated levels decreased by 1.6° at one year and although foraminal width and volume increased at six months, at one year, the width returned to baseline, and the volume was only slightly elevated. Ninety-three percent of patients had a bridging trabecular bone on CT scans performed at one year. No screws or base plates migrated although there was one partial screw backout [5]. Tan et al. reported their experience in treating 64 patients with 154 cervical levels. They found no difference in preoperative and postoperative cervical lordosis but noted that the long-term effects of these implants on fusion rates and radiculopathy remain unknown [13].

Cervical interfacet spacers are intended to treat patients with symptomatic cervical radiculopathy without symptomatic central stenosis or kyphosis. The devices are inserted through the posterior facet and abut the pedicle, which theoretically prevents plunging of the implant. Newer interfacet devices provide the theoretical advantage of a minimally invasive approach since they can be placed through a percutaneous approach. To our knowledge, this is the first report of a cervical interfacet spacer causing radiographic stenosis and clinical symptoms of non-union that were confirmed intraoperatively. Furthermore, we believe this is the first report of the removal of an interfacet spacer. Since these implants included a screw to secure the cage, removal was technically challenging and required significant removal of adjacent bone. In the absence of foraminal stenosis, it may be reasonable to treat pseudarthrosis of an interfacet spacer with supplementation by lateral mass screw fixation alone. We also present a case of interfacet implant removal due to malposition confirmed by both neurophysiologic monitoring and intraoperative CT scan. Given the positive predictive value of persistent MEP changes with postoperative deltoid palsy (67%), it is important to utilize intraoperative neuromonitoring for these cases [14].

Although early data are encouraging, interfacet spacers should be used judiciously in select patients. Intraoperative fluoroscopy may not adequately confirm implant placement, therefore we recommend consideration of intraoperative CT scan and intraoperative neuromonitoring when placing these devices. Patients with small facet joints and lateral masses (10-12 mm or smaller) may be at increased risk for malposition, thus these patients warrant careful consideration before the use of interfacet spacers. We present a retrospective, single-center study with limitations inherent to this design. Posterior cervical foraminotomy, ACDF, and total disc arthroplasty are safe and well-validated strategies for the treatment of symptomatic radiculopathy and should remain the first-line treatment. Subsequent clinical studies must compare these techniques to interfacet spacers in a prospective, randomized fashion to determine the true efficacy of the technique. For surgeons electing to use interfacet spacers, it is important to incorporate appropriate neuromonitoring techniques and intraoperative CT scans to confirm accurate implant placement.

## Conclusions

Cervical facet implants have the potential to treat radiculopathy through indirect decompression of the neural foramina, however, there are no data comparing them to well-validated procedures, including posterior cervical foraminotomy or anterior cervical discectomy and fusion. We provide the first reports of malpositioned cervical facet implants causing symptomatic foraminal stenosis. Special care must be taken when using these devices to ensure they do not violate the neural foramina. C5 appears to be particularly susceptible to postoperative deficits following implantation, and additional caution should be taken when placing C4/5 spacers. Intraoperative fluoroscopy may not adequately confirm implant placement and an intraoperative CT scan should be considered in these cases. Patients with small facet joints and lateral masses (10-12 mm or less) may be at high risk for implant malposition and warrant special consideration. Additional studies are needed to determine the long-term safety and efficacy of these devices.
